# The Current Situation and Innovation of News Communication under the Environment of Financial Media

**DOI:** 10.1155/2022/3440217

**Published:** 2022-06-18

**Authors:** Yu Wu

**Affiliations:** Media and Communications College of Weifang University, Weifang 261000, China

## Abstract

In order to solve the problem of news communication innovation in the financial media environment, meet the update needs of news communication in the financial media environment, and make up for the shortcomings of the application of emerging media technologies in news communication, it is necessary to improve people's attention to news communication. With the advent of the era of integrated media, the application of emerging media technologies such as data news and robot news to the field of news communication has shaken the status of TV news in communication and affected its news production mode, but it will not replace traditional news, become the “forced mechanism” of traditional news production reform, and boost its reform and promotion. According to the social survey of 100 people, it is found that 88 people believe that under this competition mode, the development and challenges of TV livelihood news coexist. As Yu Guoming, a professor at Renmin University of China, said, “people's livelihood news is in the process of becoming a butterfly.” TV people's livelihood news practitioners should reshape their news ideals and establish Internet thinking to face the ever-changing communication ecological environment. From channel expansion to content integration, from serving users to public opinion guidance, we are committed to building a new mainstream media with the guidance of traditional TV media, content advantages, equal communication, real-time interaction, and distinctive personality of new media. Only in this way can we obtain enough voice and influence in the highly competitive media environment.

## 1. Introduction

The development of financial media has broken the unequal relationship between traditional media communicators and audiences, and the boundaries are not as clear as before. The information between the two gradually began to flow in two directions, more of which was the relationship of cooperation and common influence. Under this background, the traditional TV people's livelihood news has also been affected. The serious loss of audience, the decreasing advertising cooperation, and the gradual reduction of viewing share are the thorny problems faced by people's livelihood news.

In his representative works “the Republic of the Internet” and “information UTO,” the famous American scholar Sonstein said that in the process of information dissemination, because the public's own information needs are not omnidirectional, the public only pay attention to what they choose and their pleasant communication field. Over time, they will shackle themselves to a “cocoon” like a cocoon. Due to the existence of “selective psychology,” users tend to contact information consistent with their own position and deliberately avoid information inconsistent with their existing position [1]. Personal choice of information has obvious tendency, without considering comprehensiveness; cling to oneness and homogeneity, and reject information of heterogeneity and diversity. In this way, the receiver will fall into the situation of self-imprisonment and self-closure, forming the “information cocoon room” effect [2]. With the advent of new media in the era of integrated media, TV livelihood news can be divided into three different stages, as shown in Figure 1.

## 2. Literature Review

Young, S. J. and others said that media integration is realized under digital technology and network technology, and the content, channel, terminal, and organization penetrate and blend with each other at different levels [3]. Different media are trying to integrate the market in terms of ownership and organizational structure while organically combining content, technology, channels, and terminals. The definition of media convergence was first put forward by Chen, Z. Its original meaning refers to the trend of multi-functional integration of various media, which is the interactive relationship between traditional media such as radio, television, newspapers, and periodicals [4]. Hazay, C. said that “media integration” in a broad sense includes the integration of all media-related media functions, means of communication, organizational structure, ownership, and other organic elements [5]. Olubiyi, I. A. believes that the “integrated media” formed by media integration is a communication concept, which is different from the disadvantages of one-way communication in the past, and transmits video, audio, text, and pictures in a variety of media [6]. Ajagekar, A. believes that different media carriers can be used to comprehensively integrate different media such as radio, television, and newspapers with common points and complementarities in terms of channel, content, and communication, so as to realize the emerging media of “resource exchange, content compatibility, mutual integration of publicity, and common prosperity of interests” [7]. Masson, E. believes that it seems that under the production cycle system of TV news programs, the host's own expression is seriously restricted and bound [8]. Zeif, R. said that news anchors broadcast more with the text content of news manuscripts and often lack the evaluative language under self-cognition [9]. Gong, X. believes that in live news programs, most news anchors are only responsible for the broadcast and reading of news manuscripts, and only a few hosts occasionally participate in the processing of manuscripts and the critical expression of personal views, which is often more true than the broadcast and reading state of manuscripts and whether the voice is fluent and smooth [10]. When news is broadcast in this way for a long time, the personal style of the news anchor is weakened, and the characteristics of the program cannot be displayed through the host's critical expression, which will also make the style of the whole program mediocre and nothing new. Because of its decision-making power to participate in a certain range of programs, the anchor system may not adapt to the situation of the news industry in the process of localization. However, we learn some of its functions, such as participating in the selection and matching of program resources and assisting the program producers in the review and modification of program content. To a certain extent, the news literacy of the anchor will be gradually improved in the working environment of the anchor system, and the overall quality of the program will also be improved in the long run.

## 3. Method

### 3.1. Internet Information Technology and Media

At present, the Internet has penetrated into all fields of people's life. The arrival of “Web 2.0” has changed people's concept of the Internet and brought users into the world of mobile Internet [11]. According to the 41st statistical report on the development of China's Internet, as of December 2017, the number of Internet news users in China had reached 647 million, with an annual growth rate of 5.4%, and the proportion of Internet users was 83.8%. Among them, the number of mobile network news users reached 620 million, accounting for 82.3% of mobile Internet users, with an annual growth rate of 8.5% [12]. As can be seen from the figure, from 3G following, 4G synchronization, and 5 g surpassing, the development of mobile Internet technology has changed the way people accept news and has also changed in the dissemination, production, and audience of TV news. The audience is more likely to receive all kinds of information, which has changed the production and broadcasting mode of TV news to a certain extent, as shown in Figures 2 and 3.

### 3.2. Analysis of Broadcast Program Content

As the trump card column of a TV station's urban channel, Watch The City has been paid special attention by the TV station. In the city channel, there is the most broadcast time every day. The broadcast time is shown in Table 1.

“Watch The City” has three live programs in the morning, middle, and evening every day. “Watch The City” morning edition is from 7 : 00 to 8 : 00 in the morning, “Watch The City” noon edition from 11 : 30 to 12 : 30, “Watch The City” evening edition from 18 : 00 to 19 : 00, and “Watch The City” Economic Life Edition from 22 : 30 to 23 : 30. The broadcast covers all aspects of people's livelihood, from the interpretation of national policies to the demands of people's life. It tells the things around people. At the same time, the source of news materials is not only the contributions of journalists, but also people can provide real-time news materials for columns through their mobile phones and other mobile terminals. The whole column is more like an information porter around the people, truly realizing the ideological line of “from the masses to the masses” [13]. In the same period of time, the audience rating of the high-frequency version is also different. The ratings ranking in recent 6 years is shown in Table 2. The viewing share in recent 6 years is shown in Table 3.

With such a high audience share, its broadcast content is more successful than other people's livelihood news columns in the city. The reason for its success is to pay attention to the proportion of people's topics in the program; pay attention to the relevant information of people in a province, such as clothing, food, housing, and transportation; pay attention to people's humanistic, emotional, and living conditions; pay attention to the decentralization of discourse power; pay attention to the speech of people in the program; express with ordinary and diversified voices; pay attention to the interaction between the program and the audience; and pay attention to the people's livelihood, life, and humanity in the broadcasting of serious news such as national events [14].

As the people's livelihood news micro-blog platform of prefecture-level municipal TV stations, the official micro-blog of “Watch The City” can develop into a new media platform with nearly 100000 within two years, with strong communication ability [15]. This is closely related to the fixed fans of the program. Among these fans, there are more fans who pay attention to 1–1.5 years and 0.5–1 years, 28.19% and 22.91%, respectively, as shown in Figure 4.

With the resource advantage of nearly 100000 fans, the official micro-blog of “Watch The City” has also become a better diffuser of people's livelihood news. At the same time, the official micro-blog maintained a high number of blogs. As of December 31, 2017, the total number of blogs of “Watch The City” was 9692, and the average daily number of blogs was about 23. Among them, the number of original microblogs is more than that of forwarded microblogs, as shown in Figure 5.

There are also fixed fan groups on various platforms. As of December 31, 2017, the number of fixed fans of “Watch The City” on the main live broadcasting platforms is shown in Table 4.

It can be seen from the above table that although each live broadcast platform has a fixed number of fans, the number of fans is not large. This problem is also the bottleneck faced by “Watch The City” in the early stage of exploring the live broadcasting platform. How to attract more fans and enhance the communication force, “Watch The City,” still needs to make greater efforts [16].

In the context of media integration, the “two sessions” report of Fujian Daily focuses on the issues most concerned by the people, making the livelihood issues closely related to the people's lives become the news theme to reflect the voice of the people. This change in communication topics not only brings the distance between the “two sessions” and the people, but also highlights the implementation of the “people's nature” principle of Fujian Daily's news publicity work, as shown in Table 5.

With the continuous development of financial media technology, the short video industry has risen rapidly and become an industrial outlet. The reasonable duration and friendly content of short video and vlog just meet the pursuit of personalization in the new media environment and meet the usage habits of new media users. It can be described as the product of Internet thinking. Local party newspapers also conform to the trend of the times, cater to the needs of the public for efficient access to information, and more in the “two sessions” news reports, choose short videos, vlog, and other forms to show the first scene of the “two sessions” news reports to the audience. At the same time, with a more daily and colloquial language style, they shorten the distance between the audience and the “two sessions.” In January 2019 to April 2020, the increment of TikTok fans is shown in Table 6.

During the “two sessions” in 2020, short videos have gradually become the leading actress in the original mobile products of Fujian Daily, “Funiu takes you to watch the two sessions,” “Shocking perspective! Experience the” ground flight “Around Fujian in two minutes!” Short video works such as “Come on, come on! Jump on a new Fujian disco” are produced from an innovative perspective, presenting the new atmosphere of the new era.

According to the latest data reported on the “two sessions” of the new Fujian app on the mobile terminal of Fujian Daily, during the “two sessions” of the province in 2020, the five platforms on the mobile terminal of Fujian Daily worked in the same direction and published about 310 relevant reports in eight days from the 9th to the 16th [17]. Among them, the new Fujian client has about 180 copies, 21 WeChat releases, 42 micro-blog releases, 53 TikTok releases today, and 13 videos [18] with small video. The number of reports from different platforms of Fujian Daily from 2014 to 2019 is shown in Table 7.

### 3.3. Rationalization Evaluation and Analysis of Network News Communication Effect Prior Data Sampling and Statistical Analysis

In order to realize the accurate evaluation of the rationalization evaluation of network news communication effect, a priori data collection of the rationalization evaluation of network news communication effect is carried out by using the methods of big data analysis and quantitative evaluation of statistical characteristics. It is assumed that the prior knowledge of time series sampling of statistical network news communication effect rationalization evaluation data is expressed as {*xi*}. Arrange the quantitative distribution data of network news communication effect according to the feature set of sequence *y* '(*n*), and obtain the original sequence of rationalization evaluation of network news communication effect, as shown in formula (1). Using the adaptive regression analysis method to construct the characteristic component of the rationalization evaluation data of network news communication effect, study the rationalization evaluation model of network news communication effect, divide the rationalization level of network news communication effect into N levels, and obtain the adjustment model of rationalization evaluation of network news communication effect, as shown in formula (2), formula (3), formula (4), and formula (5).

(1) $$\begin{array}{c} \left\{\varsigma xi\left(jk\right)\right\}=xjk-xi. \end{array}$$

(2) $$\begin{array}{c} \text{min}F=R^{2}+A\sum_{i}\xi i. \end{array}$$

(3) $$\begin{array}{c} \text{s}.\text{t}:{\left\|\phi \left(xi\right)-0\right\|}^{2}. \end{array}$$

(4) $$\begin{array}{c} \text{max}\sum_{i}aik\left(xi,xi\right)-\sum_{i}\sum_{j}aiajK\left(xi,xj\right)\sqrt{a^{2}+b^{2}}. \end{array}$$

(5) $$\begin{array}{c} \text{s}.\text{t}:\sum_{i}ai=1. \end{array}$$

The above formula is expressed as a normal distribution function. *O* is the inertia weight of the statistical characteristic distribution of the network news communication effect. Considering the statistical characteristic prediction value of the rationalization evaluation of the network news communication effect, the factor analysis of the rationalization evaluation of the network news communication effect is carried out in combination with the multivariate linear fusion method. The load of data sampling is shown in

(6) $$\begin{array}{c} B_{N\times 1}=S_{N\times L}•T_{L\times 1}. \end{array}$$

Through autocorrelation feature matching, the statistical features of the rationalization evaluation of network news communication effect are obtained. There is a mapping relationship between the predicted nonlinear statistical features *RN* and *XN*, as shown in

(7) $$\begin{array}{c} p\left(R^{N}=ri\right)=P\left(X^{N}=xi\right). \end{array}$$

(8) $$\begin{array}{c} p\left(R^{N}=ri\right)=P\left(\text{angle}\left(ri\right)-\phi g\right)\text{mod}\left(2\pi \right). \end{array}$$

The statistical average analysis method is used to construct the big data model for the rationalization evaluation of network news communication effect, and the descriptive statistical analysis method is used for the positive correlation analysis of the sampled big data. The mutual information transfer function description of the rationalization evaluation of network news communication effect is shown in

(9) $$\begin{array}{c} I\left(X^{N};Z^{N}\right)=H\left(X^{N}\right)-H\left(X^{N}|Z^{N}\right). \end{array}$$

(10) $$\begin{array}{c} ?=H\left(X^{N}\right)-H\left(X^{N}|Z^{N}\right)-H\left(\phi G|Z^{N}\right). \end{array}$$

When the effect of network news communication is rationalized, the number of iterations *V* of quantitative recursive analysis of statistical big data is the minimum. When *VVT* = *IM* has a minimum value, set the value of inertia weight *o* for propagation effectiveness evaluation, as shown in formula (11).

(11) $$\begin{array}{c} w=w\text{max}-t\frac{w\text{max}-w\text{min}}{T\text{max}}. \end{array}$$

*W*max and *W*min, respectively, represent the regulation coefficient of the rationalization evaluation of network news communication effect, *T*max is the maximum control time scale, and *t* is the random number of hops of the rationalization evaluation of network news communication effect. In the vector space of *m* dimension, the statistical characteristics of the rationalization evaluation of network news communication effect are analyzed, and the statistical model is obtained, as shown in

(12) $$\begin{array}{c} w=w\left(t\right)*w\text{start.} \end{array}$$

(13) $$\begin{array}{c} w=w\left(t\right)*\frac{1}{w\text{end}}. \end{array}$$

The vector quantization decomposition of media factors is carried out by linear exponential analysis method, and the decomposition form is shown in

(14) $$\begin{array}{c} \text{s}.\text{t}\sum_{\left(i,j\right)\subseteq E}gij-\sum_{j\subseteq V}gji. \end{array}$$

(15) $$\begin{array}{c} \sum_{\left(j,i\right)\subseteq E}g^{e}ji=T\theta_{i}^{e}. \end{array}$$

Use ▲*Mij* (*i* = 1, *D*; *j* = 1, *N*) to represent the contribution of the rationalization evaluation of network news communication effect. Combined with the descriptive statistical analysis method, the related factor modeling of the rationalization evaluation of network news communication effect is realized [19].

To some extent, the impact of the new media era on the traditional TV media is devastating. If we cannot find ways and methods to move forward together in the multi-channel of media integration, the limitations of traditional media communication methods and effects will inevitably affect our own development and progress in a long time. Therefore, TV people's livelihood news should continuously and deeply explore the communication effect after media integration in the process of media integration, so as to ensure that the TV people's livelihood news after media integration can maintain lasting program vitality under the new media integration environment [20].

Media environment is a social situation, which includes all factors that may affect the development of media. The concept of media environment originated in the 1960s and was put forward by Canadian communication scientist Marshall McLuhan [21]. This makes the initial media environment defined as the expression of a social situation. Media environment is a social situation, which includes all factors that may affect the development of media. Then, according to Posman's definition of media environmentology, “media environmentology studies human communication, the information and information system of human communication. Specifically, media environmentology studies how the media affects people's perception, emotion, cognition and value, and how our interaction with the media promotes or hinders our chances of survival.” Under the background of the rapid development of media integration, TV people's livelihood news needs to clarify ideas, find appropriate methods to conduct in-depth exploration, and grow and progress in a new media environment [22].

TV people's livelihood news always adheres to the principle of “content as the soil” to produce and build programs. However, in the face of the impact of new media, the TV livelihood news program with the original content of “trump card” is facing the disadvantages that the timeliness of program resources is not as fast as network media in the environment of new media. In the face of the media environment of financial media innovation, the traditional TV media has also changed to the strong position of information resource provider in Japan. Now we also need to face the transformation of the way of supplying program information together with the new media on the Internet [23]. First of all, we need to make it clear that the branding of TV livelihood programs is a prerequisite to ensure that TV programs can get a share in the all media era when they are kidnapped by ratings. Today's TV media providers, under the overall situation of the integration of new media, in addition to the high-quality guarantee of self-made news programs, the video forwarding of the official WeChat public platform of the program, and the sharing and interaction of program micro-blog should also ensure the overall awareness of high-quality programs. Only by ensuring the quality of program content and packaging, the ratings and advertising sponsorship of TV livelihood news programs can maintain stable development to a certain extent [24].

According to Philip Kotler, an American marketer, “a brand is a name, term, symbol or pattern, or a combination of them, which is used to identify the products or services of a seller or a group of consumers and distinguish them from the products or services of competitors.” Brand is a concept in marketing, but it also plays a great value in the development and layout of the TV media market. Just like in daily life, we buy different goods in supermarkets according to our own understanding of brands. The branding strategy of TV livelihood news programs is to strive for high returns from advertising sponsors and the audience's conventional qualitative thinking means for program experience [25]. For example, Zhejiang Radio and television station have positioned its own satellite TV channel as “China Blue—the first dream channel.” According to the theme of the dream, it has created a variety show “China Dream Show” to help ordinary people realize their dreams. According to its own brand strategy, it attracts the sponsorship of advertisers, so as to promote the balanced development of other TV programs on the channel. TV people's livelihood news should also learn to optimize the “trump card” of its own programs, so as to achieve the brand strategy of ensuring the rapid development of programs. The strategic way of transitioning from programs to successful brand programs also needs to mature under the influence of program arrangement, innovation, brand power, publicity, and competitiveness [26], as shown in Figure 6.

At present, the integration of traditional media and new media is still running in and adapting to each other. For TV news programs with high brand value, trying more brand-new interactive experiential activities will give loyal viewers a higher degree of program loyalty and satisfaction. It is nothing more than an exploratory attempt to transform the audience from a single audience who pays attention to the people's livelihood news of TV programs to consumers who trust the brand credibility of TV programs. This is also a successful TV news program. From the acquisition of information focusing on people's livelihood to the secondary dissemination of people's livelihood information based on the power of brands, it can deeply explore the competitiveness of program brands [27].

Young TV audiences are more likely to participate in the online and offline brand interaction experience of the program through the dissemination of new media. In the interactive process of the column group, the satisfaction of the audience and the sense of existence of the program are greatly increased, and a good activity experience is obtained in the program. Then, in the offline communication process of the brand program, the column group itself should pay more attention to the brand derivative communication effect of the program, bring good user experience to consumers, and then ensure the legitimate rights and interests of consumers.

For the in-depth exploration of media integration, we need to further deepen the in-depth expression of communication influence. The people-friendly characteristics of TV people's livelihood news are incomparable advantages of other types of news, but we should also be aware of how to have a strong objective and fair perspective in the process of news reporting in addition to being considerate of the people's suffering. This also puts forward new improvement ideas for the people's livelihood TV news under the background of new media, because the host broadcasting type of TV people's livelihood news programs is mostly the popular “say” news in recent years, which has stimulated the audience's interest in watching. However, we should also think about whether the people-friendly “say” news has broken the fairness and authority of the news. Therefore, in the report of TV people's livelihood news, we should also pay attention to the richness and diversity of topics, and avoid repeated and typed life trivia, because to a certain extent, it will also make the audience cause aesthetic fatigue in the viewing process, and it is difficult to become a brand name program in the evolution process of program form.

With the development of information processing, storage and transmission technology, and the low threshold of information production, a large amount of information is increasingly flooded in the Internet. In the context of massive, quantitative, and even astronomical information, users' attention has become an extremely scarce resource. From the perspective of users, it is extremely laborious to obtain valuable information for their own use from a large amount of information. From the producers and disseminators of information, how to make their information stand out and be noticed by target users has become extremely important. In this context, TV people's livelihood news is also actively rewriting the news production and broadcasting mechanism of traditional media. They have imitated the trump livelihood programs with successful communication effects, copied their news types, host styles, and broadcast time, and actively sought innovative ways, but also brought many new problems.

## 4. Results and Analysis

Facing the current situation of changing the communication mode of TV people's livelihood news, we should learn about the publicity and improvement of media marketing. Traditional enterprises rely on newspapers, radio, and television to carry out commodity publicity. When new media rise, it has changed quietly. A large number of enterprises have gradually reduced their original advertising investment in television, radio, and paper media, and then occupied the Internet market. In the face of the current situation that its advertising sponsors turn to other media for marketing and publicity, on the premise of good quality of its own programs, the TV people's livelihood news program also tries to attract other enterprises that need advertising and publicity to invest and sponsor according to the competitiveness of its own programs, strive for local enterprise advertising resources, and do a good job in offline audience interactive experience activities to enhance the vitality of the program so that viewers who pay attention to the program can be closer to the program, and it is also convenient for potential advertisers to observe and think. In this way, it also alleviates the dilemma of the lack of sponsored advertisers for the livelihood news programs on the ground channel to a certain extent. In addition to the offline activities to promote advertisers, the team members of the TV people's livelihood program group can also plan the online sponsor product exhibition and marketing, relying on the column's own brand influence to market the sponsor advertising products on the network, so as to achieve the virtual environment profit model of advertisers for market publicity.

When the communication mode of traditional media is facing the process of integration with new media, the traditional concept should also be updated in time. The current TV content supply platform transmits more different types of fresh TV news information to the audience. Under the new media pattern with Internet terminals, the traditional media should realize that the content released by themselves will be given to the audience through different media, and today's TV audience has also transitioned from the traditional TV audience to the all media user. This also determines that the information based on the content platform can be spread to more users through more diversified communication channels such as websites, publications, and radio.

In the face of TV livelihood news programs under the condition of industrial chain, we need to appropriately adjust the structure of our own programs, screen the “gold content” of program content, and pay more attention to the “big news” of people's livelihood. Find typical news from “small stories” and dig more in-depth reports of news. When a variety of media methods compete for the attention of audience users, the perspective and depth of news reporting determine the position of TV people's livelihood news in competition with other media. If we care about each other with the content on the new media platform, TV Minsheng news will be truly recognized by the audience with its own depth and reporting rigor. However, if the audience wants to get fresh first-hand news information, new media has become the best choice because of its faster communication speed. News websites on the Internet, mobile app news clients, and news on micro-blog and WeChat are transmitting the content of news information from their own perspectives. Therefore, facing the traditional TV news media in the multi-angle industrial chain, people should adapt to their respective advantages and their own positioning in the integrated media environment and strengthen their own livelihood perspective news. Even in the integration process, they cannot blindly cater to the communication mode of new media. If the traditional TV media loses its own news attribute in the integration process, it will eventually be “shuffled” and eliminated in the process of media reform. Therefore, in the process of integration, we should learn the complementary advantages of media and learn to explore new ways of reporting in a timely manner. Under the new normal Internet plus media era, we will try to find a new look of TV news about people's livelihood in the background of new media convergence.

At present, the columns of TV people's livelihood news basically meet the needs of middle-aged and elderly audiences, such as life services, daily conversation, and curiosity. This is because practitioners believe that local middle-aged and elderly TV viewers mainly watch livelihood news. In the fixed demographic dividend, the inherent personality endorsement has been formed. The result of this vicious circle is that while it cannot attract new audiences, it will lose the fixed audience transferred to other new media due to fatigue and curiosity at any time. Such a development has a devastating impact on TV people's livelihood news. To enhance the vitality of people's livelihood news in the media era and attract young audiences from different groups is the only way out for TV people's livelihood news. The way for young people to receive news is mainly through the Internet and mobile terminals. Therefore, cultivating young audiences is also the only way for TV media to develop financial media communication.

To cultivate young audiences, we must first rebuild the vitality of people's livelihood news. Use professional news to record the most important things around local people. In terms of news content, we should strictly screen news topics with social value and application value. Meet the needs and habits of young people, such as employment information suitable for college students, housing information suitable for young people entering the workplace, and parenting information suitable for young mothers. In terms of communication voice, news language should be more fashionable and interesting.

## 5. Conclusion

Speed up the combination of TV people's livelihood news and financial media, and establish all-round employees in the workflow. Journalists should have all-round media ability and high ideological and cultural literacy, and master the live broadcasting process of traditional media and the use of mobile media equipment. Everyone in the team has the ability to skillfully use multiple media. After getting the livelihood news, the collected content can be transmitted to different broadcasting platforms such as TV, network, and mobile terminal as soon as possible, and presented to the audience in different ways such as text, picture, video, and audio. All media editors can not only give full play to their own expertise to complete the new media editing work alone, but also flow across posts and give full play to their post-responsibilities in the overall operation. With good teamwork spirit, media integration awareness, innovative spirit, and professional quality, it is a necessary quality for “one specialty and multiple abilities” all media editing talents. Through the data analysis of “Watch The City” and “Fujian Daily,” it is proved that it is very important to understand and solve the problem of news communication innovation in the financial media environment. It can effectively solve the problem of insufficient application of emerging media technology to news communication, meet people's demand for the emerging of news communication, make up for the insufficient application of emerging media technology to news communication, and improve people's attention to news.

## Figures and Tables

**Figure 1:** Development process of people's livelihood news.

**Figure 2:** China's online news users in 2016.

**Figure 3:** China's online news users in 2017.

**Figure 4:** Analysis of the number of years of attention of fans on the official micro-blog of “Watch The City.”

**Figure 5:** Proportion between the number of original microblogs and the number of forwarded microblogs of the official micro-blog of “Watch The City.”

**Figure 6:** “Fishbone” strategy of program branding.

**Table 1:** Daily broadcast time period of “Watch The City.”

Playback period	The name of the “Watch The City” column in different time periods
07 : 00--08 : 00	“Watch The City” morning edition (live broadcast)
11 : 30--12 : 30	“Watch The City” midday edition (live broadcast)
18 : 00--19 : 29	“Watch The City” evening edition (live broadcast)
22 : 30--23 : 30	“Watch The City” (Economic Life Edition)

**Table 2:** Ratings ranking of “Watch The City” in recent 6 years.

Column	2013	2014	2015	2016	2017	2018
“Watch The City” morning edition	1	2	7	8	3	3
“Watch The City” midday edition	17	22	10	40	12	10
“Watch The City” evening edition	1	1	1	1	1	1
“Watch The City” (Economic Life Edition)	18	19	37	14	25	31

**Table 3:** Ranking of audience share of “Watch The City” in recent 6 years.

Column	2013	2014	2015	2016	2017	2018
“Watch The City” morning edition	11.21	12.55	5.71	3.88	7.01	8.44
“Watch The City” midday edition	2.31	2.01	2.94	0.55	2.71	4.08
“Watch The City” evening edition	20.11	19.04	14.77	13.49	15.88	15.62
“Watch The City” (Economic Life Edition)	1.19	1.81	0.23	2.66	0.11	0.51

**Table 4:** Number of fans on the live broadcast platform of “Watch The City.”

Program name	Yingke live broadcast	Panda live broadcast	Pepper direct seeding	Youku live
Number of fans	857	524	498	377

**Table 5:** Number of reports on different types of topics in Fujian Daily from 2014 to 2019.

Topic type	Media type					
	Newspaper	Official account	Client	Micro-blog	Total	Proportion (%)
Politics	397	21	10	64	471	56.20
Economics	134	9	3	32	169	20.17
People's livelihood	104	3	2	13	119	14.20
Ecology	43	1	1	6	50	6.0
Legality	23	0	0	6	29	3.5
Total	701	34	16	121	838	—

**Table 6:** The increase of TikTok fans in one year from April 2019 to April 2020.

Date	2019.1	2019.4	2019.7	2019.10	2020.1	2020.4
Fans growth	11	49	79	134	143	155

**Table 7:** Number of reports on different platforms of Fujian Daily from 2014 to 2019.

Particular year	Newspaper	Official account	Micro-blog	Client	Total
2014	120	0	2	0	122
2015	120	7	2	0	122
2016	119	6	4	0	123
2017	120	1	18	2	140
2018	118	2	38	8	164
2019	106	18	56	5	167
Total	703	34	120	15	838

## Data Availability

The labeled data set used to support the findings of this study is available from the author upon request.
